# How Different Motivations for Making Informal Out-Of-Pocket Payments Vary in Their Influence on Users' Satisfaction with Healthcare, Local and National Government, and Satisfaction with Life?

**DOI:** 10.1155/2021/5763003

**Published:** 2021-08-26

**Authors:** Nazim Habibov, Alena Auchynnikava, Lida Fan, Yunhong Lyu

**Affiliations:** ^1^School of Social Work, University of Windsor, 167 Ferry Street, Windsor, Ontario, Canada N9A0C5; ^2^University of Windsor, Ontario, Canada; ^3^Lakehead University, Thunder Bay, Ontario, Canada

## Abstract

**Background:**

The dominant view in the literature is that informal payments in healthcare universally are a negative phenomenon. By contrast, we theorize that the motivation healthcare users for making informal payments (IP) can be classified into three categories: (1) a cultural norm, (2) “grease the wheels” payments if users offered to pay to get better services, and (3) “sand the wheels” payments if users were asked to pay by healthcare personnel or felt that payments were expected. We further hypothesize that these three categories of payments are differently associated with a user's outcomes, namely, satisfaction with healthcare, local and national government, satisfaction with life, and satisfaction with life of children in the future.

**Methods:**

We used microdata from the 2016 Life-in-Transition survey. Multivariate regression analysis is used to quantify relationships between these categories of payments and users' outcomes.

**Results:**

Payments that are the result of cultural norms are associated with better outcomes. On the contrary, “sand the wheel” payments are associated with worse outcomes. We find no association between making “grease the wheels” payments and outcomes.

**Conclusions:**

This is the first paper which evaluates association between three different categories of informal payments with a wide range of users' outcomes on a diverse sample of countries. Focusing on informal payments in general, rather than explicitly examining specific motivations, obscures the true outcomes of making IP. It is important to distinguish between three different motivations for informal payment, namely, cultural norms, “grease the wheels,” and “sand the wheels” since they have varying associations with user outcomes. From a policy making standpoint, variation in the links between different motivations for making IP and measures of satisfaction suggest that decision-makers should put their primary focus on situations where IP are explicitly asked for or are implied by the situation and that they should differentiate this from cases of gratitude payments. If such measures are not implemented, then policy makers may unintentionally ban the behaviour that is linked with increased satisfaction with healthcare, government, and life (i.e., paying gratitude).

## 1. Background

IP is defined as a direct contribution in cash or gifts that is in addition to any formally required contributions and which are made by users to healthcare personnel or others acting on their behalf [1, 2]. Since such payments are made out of the counter and under the table, they are not part of formal healthcare expenditures and can be made in the form of cash such as small tips and large sums of money, or through various types of gifts such as flowers and sweets, and before or after receiving services [3]. IP is a subsection of a wider category of out-of-pocket payments [4]. Thus, out-of-pocket payments represent the amount of IP and legitimate legal fees paid in the healthcare sector taken together. Legitimate fees may include copayments for compulsory and voluntary health insurance schemes and payments for healthcare services which are not covered by compulsory and voluntary health insurance schemes.

Various estimates show that IP represents the lion's share of out-of-pocket payments [5]. For instance, the share of IP has reached 96% in Pakistan [6] and 74% in Azerbaijan [7]. Even in EU and OECD countries, incidents of IP are high, reaching 35% in Poland, 41% in Lithuania, and 17% in the Czech Republic and Slovakia [7]. From the standpoint of health policy and planning, such a large share of IP underlines a shift in healthcare funding from a solidarity approach that is based on budget-financed or insurance-financed schemes, to an individualistic approach where consumers are expected to bear the main responsibility for healthcare costs [8, 9].

Against this background, the literature highlights a lack of studies on association between different motivations for IP and user outcomes and points out that the current literature tends to evaluate overall effect of IP without considering different motivations for making IP [10, 11]. With the above evidence in mind, we theorize that the motivations for making could be grouped into three broad categories, namely, “cultural norm,” “grease the wheels,” and “sand the wheels.” We further theorize that the direction of association between IP and satisfaction is not universal and depends on the specific motivation for making IP. More specifically, we hypothesize that “cultural norm” and the “grease the wheels” conceptualization of IP may be associated with positive user outcomes, while the “sand the wheels” conceptualization will have an opposite association. To test these hypotheses, we separately analyze the effect of each of the above-discussed theoretical motivations of IP on user well-being. This approach allows us to shed light on differences in the association between the various motivations for making IP with a wide range of users' outcomes. In this way, the study answered to the following three research questions:

1. How do each of these motivations influence satisfaction with public healthcare?
2. How do each of these motivations influence satisfaction with local and national governments?
3. How do each of these motivations influence satisfaction with one's own life and expected satisfaction with the future life of one's children?

The unique contribution of this study is threefold. First, as far as we know, this is the first study which tests for plausible variation in the influence of the different conceptualizations of IP on users' outcomes on a large sample of countries. Second, we test for the influence of IP on a wide range of outcomes including satisfaction with local and national governments and satisfaction with one's own life and expected satisfaction with the future life of one's children.

Finally, we focused on postcommunist countries where incidents of IP are high and have a prolonged history. Historically, under the Semashko system, the state in the communist countries assumes the primary responsibility to provide universal healthcare to the citizens free at the point of utilization [12]. However, considerable shortage in the available public funding together with the nonexistence of official and legitimate mechanisms for engaging private healthcare expenditures led to widespread inequalities in access in the 1970s and IP became an important factor in ensuring access to rationed public healthcare since 1970s [13, 14]. The role of IP in providing access to public healthcare further grew through 1980 as postcommunist countries were not able to sufficiently increase public finding for healthcare and IP became widespread in forms of cash and small gifts, for instance, liquors, cigarettes, and perfume [15–17]. Collapse of communist economic system in the 1990s increased the spread of IP since the profound and protracted political and economic crisis associated with transition from communist further reduced public funding for healthcare [18, 19].

To curb IP, postcommunist countries embraced the wide range of healthcare reforms and each postcommunist country has chosen their own way for reforms with at least four main models were utilized: (1) to introduce compulsory health insurance system, (2) to implement guaranteed benefit packages for specific types of healthcare services or for specific population groups (e.g., maternal healthcare and healthcare for internally displaced people), (3) to use some combination of both above-described approaches, and (4) to remain with a traditional model of healthcare financing where healthcare funding is paid from the general budget revenue [20–23]. The fully comparable data about current characteristics of the healthcare systems in postcommunist countries is hard to find, so Table 1 provides the available information from the Global Health Expenditure database by the WHO that is the most reputable source of cross-country comparison for healthcare [24].

The reforms were not able to substantially reduce incidents of IP in postcommunist countries [25–27]. The recent studies conducted after 2010 reveal that incidents of making IP remain widespread. Thus, Stepurko et al. [25] found that the scale of making IP in forms of gifts varies from 35 percent in Poland to 58 percent in Ukraine. The most recently available estimates for postcommunist countries show that IP is considerable not only in low-income countries, for instance, 74 percent in Azerbaijan and 65 percent in Kyrgyzstan, but also in high-income countries, for instance, 34 percent in Hungary and 44% in Romania [7]. The literature indicates multiple interrelated reasons why IP were not significantly reduced as a result of the reforms. First, population health worsened because of depression, stress, ethnic wars, civil and political conflicts, corruption, and crime which are associated with the period of the transition from communism [28–30]. In turn, the worsening health increased demand for healthcare. Second, the reforms were not able to substitute the considerable deficit of public healthcare financing which happened during the transition [25]. Third, expectations of users about quality of healthcare continued to increase substantially during the transition and making IP was often considered the only way to gain access to higher quality and faster healthcare [10, 31]. Finally, many healthcare users felt that the state ceased to be responsible for their health and they must use all available ways to get access to healthcare including making IP [32].

## 2. Materials and Methods

### 2.1. Main Theoretical Argument: Three Motivations for IP and Their Links with Users' Outcomes

One the most accepted schools of thought conceptualizes IP as a cultural phenomenon that originates in the social norms of gratitude. According to this approach, users, healthcare personnel, and health administrators argue that cash payments or gifts given by healthcare users to healthcare personnel are consistent with customs and traditions that are rooted in cultural norms and beliefs of gift giving and reciprocity [33–35]. The notion of IP as a cultural norm of gratitude is asserted to be particularly relevant to nations outside of the realm of Western culture and tradition [36–38]. As justified by Yang [39], incidents of IP “cannot be reduced to a modern western notion of corruption because the personalistic qualities of obligation, indebtedness, and reciprocity are just as important as transactions in material benefit.” Thus, although large-scale corruption schemes in public services, and especially in healthcare, are commonly criticized, IP given to healthcare personnel are not necessarily considered to be the result of illegal corruption [40–43]. The important implication of conceptualizing IP as a non-0 form of gratitude payment is that there will be a positive association between making IP and a higher level of satisfaction and well-being for users who have paid IP. Thus, the following hypotheses can be articulated based on the discussion above:

*H1 Gratitude motivation for making IP is associated with a positive user's outcomes.*

Another school of thought conceptualizes IP as a “grease the wheels” phenomenon and suggests that IP can alleviate the limitations of the healthcare system including its slow speed of action, low quality, and the competition between providers of public services in less-developed countries [11, 44]. It posits that users' primary motivation for making IP is the prospect that they will receive a quicker and a higher quality of care that is more personalized and convenient and has shorter wait times and that they will have access to more advanced or specialized care and services [2, 45–47]. As an illustration, Riewpaiboon and colleagues detailed how a Thai woman made informal payments to an obstetrician to get better services during her pregnancy [48], while several other studies confirmed that IP resulted in a better relationship between users and healthcare personnel and consequently in higher levels of satisfaction for users [4, 5, 49, 50]. On the other hand, IP eases the inefficiencies of administering public healthcare in a situation where healthcare workers believe that they are not being paid adequately and so have the expectation of IP, while concurrently, users expect to pay out-of-pocket to underpaid professionals for more or better-quality service [15, 41, 51, 52]. As such, when the expectations of healthcare professionals and the users of healthcare are congruent; then a transaction between the payment and reception of unofficial payments takes place. Furthermore, IP could encourage competition between healthcare providers and could be financially beneficial for users. Thus, it could occur that users would need to pay less IP for formally “free” treatment in public healthcare rather than to officially pay more for the same treatment in private healthcare [7, 53]. The “grease the wheels” conceptualization suggests a statistically significant association between making IP and positive users' outcomes. Consequently, our next hypothesis is

*H2 “Grease the wheels” motivation for making IP is associated with a positive user's outcomes.*

The last school of thought conceptualizes IP as the more negative “sand the wheels” phenomenon and highlights that the above-discussed perspectives are used to normalize IP in healthcare and make an unacceptable phenomenon acceptable [1]. It posits that users have to make IP since they are directly asked by healthcare personnel or they know that such payment is expected, while not making IP will negatively affect access to services or the quality of the services they receive [8, 10, 25, 54]. As an example, Miller et al. [55] (p. 310) cited a respondent in Bulgaria who described the fate of another user's father “He [son of another user] was told he had to give 20,000 levs. He said he could afford only 10,000 levs. And two days later his father died.” Furthermore, another respondent in the Ukraine emphasized, “When the matter has to do with health, you go ahead and give bribes. Health is more important than anything.” Another of the negative impact of IP includes a decrease in the likelihood of using healthcare when needed, in particular for the poor for whom IP frequently represents catastrophic expenditures [56–59]. Equally, IP is a serious barrier for access to more advanced and specialized types of treatment [60, 61]. The “sand the wheels” conceptualization of IP suggests a significant negative association between IP and user outcomes. Thus, our final hypothesis is

*H3 “Sand the wheels” motivation for making IP is associated with a negative user's outcomes.*

### 2.2. Data

We followed the methods of Habibov et al. [62]. Our study is based on the secondary analysis of microdata from the 2016 Life-in-Transition survey (henceforth, the LITS) that covers 27 postcommunist countries of Eastern Europe and the former Soviet Union. The LITS was implemented by the Ipsos pollster company with support from the European Bank for Reconstruction and Development and the World Bank [63]. The survey collects information about IP in each country and about the socioeconomic characteristics of respondents and their households.

The LITS employs a multistage design. The survey employs the list of primary selection units (PSUs) which is derived from the most recent sample frames prepared by the countries' national statistical organizations in the first stage of sampling. The probability proportional to size technique is employed to choose the PSUs from the frames in the second stage of sampling. In this way, depending on the size of the country and its population density, approximately 50-70 PSUs in each country are selected for surveying. During the third stage, the random walk technique is used to choose households for interview in each of the selected PSU. In the case where more than one household lives at the same address, then only one of the households was randomly selected to participate in the survey. During the final stage, one household member was selected for an interview using the last birthday technique. Up to three home visits were conducted to heighten the chances that the chosen respondents would be able to participate in the survey. Specially trained investigators then interviewed approximately 1000 respondents in each country under investigation, with an overall response rate of 89%.

The original English version of the master questionnaire was developed in conjunction by Ipsos, the EBRD, and the World Bank. It was then translated into the local languages by experienced professional interpreters. In translation, the questionnaire was then sent to each country to be checked and approved by local interviewers and agencies. Feedback from each country was then given to professional translators who rechecked the translated national versions. All the suggestions for adjustments made by the local teams were incorporated into the final version of the survey. In countries where Russian is spoken, survey participants were given the option of using the Russian version. After the questionnaire was pretested, suggestions were again incorporated into the questionnaire. The amended version of the questionnaire was then used for the pilot that was conducted in each country by local interviewers and agencies. Criticism and advice resulting from these pilots occasioned additional changes to the questionnaire.

### 2.3. Definitions and Measurement

Detailed description of all the variables including descriptive statistics can be seen in Table 1, while further discussion of the descriptive results can be found in Figure 1. As such, here, we will confine ourselves to a brief outline of the variables used in this study. We commence with making IP. The LITS asked each respondent who had used the healthcare system within the last 12 months whether she or he had “made unofficial payments or gifts (with the exception of any official fees or payments) during the last 12 months.” The response is recorded as binary (yes = 1; no = 0). The same definition of IP has been used in previous studies [7].

Next, respondents who had made IP were asked about their motivations for doing so. We conceptualized IP payment as a “grease the wheel” payment if the respondent had indicated that they had offered to pay IP to get better or quicker services. In contrast, we conceptualized it as a “sand the wheel” payment if the respondent indicated that IP was made because they had been asked to pay it by healthcare personnel or felt that IP was expected. Lastly, if the respondent reported making IP to express customary gratitude to healthcare personnel, it was considered a “gratitude payment.” All motivation variables are recorded as binary (made a specific type of IP = 1; no = 0).

The LITS allows us to distinguish between four types of users' outcomes, namely, satisfaction with healthcare, local and national government, satisfaction with life, and satisfaction with life of children in the future. All variables are ordered Likert-scale variables ranging from 1 to 5, where a higher value indicates a more satisfaction.

### 2.4. Analytic Approach

We regress making IP on satisfaction with healthcare, local and national government, satisfaction with life, and satisfaction with the anticipated future life of one's children. We estimate a series of ordered logit regressions since satisfaction is measured by ordered Likert-scale type variables. All regression models controlled for covariates that are typically associated with making IP including individual-level characteristics such as age, gender, education, marital status, self-assessed health status, and household-level characteristics such as number of young and older children, household wealth, and residing in rural areas [7, 8, 25]. To control for country-level differences, all models included country dummies. To control for PSU influence, all models include cluster-robust standard errors. All models reported odds ratios, standard errors, and statistical significance at conventional levels (^∗^*p* < 0.05, ^∗∗^*p* < 0.01, and ^∗∗∗^*p* < 0.001).

## 3. Results

### 3.1. Descriptive Results

Descriptive results for main predictor of interest are reported in Figure 1, which illustrates the flow chart of the IP-related questions. As shown, approximately 18% of respondents made IP. Among those who made IP, about 31% did so to express gratitude. In contrast, about 19% offered to pay to get better services. However, the largest share of respondents who made payments, approximately 45%, were asked to do so by healthcare personnel or felt that IP were expected.

Further descriptive results for IP payments are reported in Table 2. This table shows the percentage of respondents who reported to make IP in each country. Among countries of the former Soviet Union, respondents from Tajikistan, Moldova, and Azerbaijan reported the highest incidents of making IP—46, 42, and 35 percent, respectively. The lowest number of IP incidents in the countries of the former Soviet Union is reported in Georgia (3 percent) and Uzbekistan (16 percent). Looking at the postcommunist countries of South Europe, we can find that highest proportion of respondents paid IP in Albania 31 percent and Romania 30 percent. The lowest percentage of IP in South Europe can be observed in Croatia (9 percent) following by Macedonia (10 percent). Remarkably, IP are widespread in more developed postcommunist countries of Eastern Europe such as Hungary with 25 percent and Lithuania with 24 percent. Approximately 13 percent of respondents reported paying IP in Slovakia and 12 in Latvia. The lowest incidents of making IP in Eastern Europe can be found Slovenia (2 percent) and Estonia (5 percent).

Finally, a sociodemographic and economic description of the analytical sample is presented in Table 3.

### 3.2. Influence of IP Motivations on Satisfaction with Healthcare

We begin with examining the association between motivations for providing IP and satisfaction with healthcare. The results of ordered logit regressions on satisfaction with healthcare are reported in Table 4. Overall, as shown in Model 1, making IP is associated with a significant reduction in the likelihood of reporting satisfaction with healthcare. However, results of Models 2 to 4 show that the association between IP and healthcare satisfaction depends substantially on one's specific motivations for making IP. Thus, the results of Model 2 suggest that making IP as a cultural norm of gratitude is associated with increased satisfaction with healthcare. In comparison, results of Model 3 indicate that offering to pay IP in order to get better service (i.e., the “grease the wheels” conceptualization) is not significantly associated with healthcare satisfaction. To the contrary, results of Model 4 signal that paying IP because it is expected or asked for (i.e., the “sand the wheels” conceptualization) significantly reduces satisfaction with healthcare.

### 3.3. Influence of IP Motivations on Satisfaction with Local and National Governments

We proceed with evaluating the relationship between IP and satisfaction with local and national governments. The results of ordered logit regressions on IP on satisfaction with local government are reported in Models 5 to 8 of Table 5. Overall, as shown in Model 5, making IP is associated with a significant reduction in the likelihood of reporting higher satisfaction with local government. Nevertheless, the association between IP and healthcare satisfaction varies considerably across specific motivations for making IP. Indeed, paying IP because it is a cultural norm of gratitude significantly increases satisfaction with local government in Model 6. In contrast, offering to pay IP in order to get better service (i.e., the “grease the wheels” conceptualization) is not significantly associated with satisfaction with local government in Model 7. Finally, making IP because it is expected or asked for (i.e., the “sand the wheels” conceptualization) is associated with a reduction in satisfaction with local government in Model 8.

The results of ordered logit regressions on IP on satisfaction with national government are reported in Models 9 to 12 of Table 4. Making IP overall in Model 9 is associated with a significant reduction in the likelihood of reporting satisfaction with the national government. Nonetheless, in the line with our previous results, the association between IP and healthcare satisfaction varies across specific motivations for making IP. Hence, Model 10 suggests that having made IP as a customary show of gratitude significantly increased satisfaction with the national government. Conversely, making IP because it is expected or asked for (i.e., the “sand the wheels” conceptualization) significantly reduced satisfaction with the national government in Model 12. In contrast, offering to pay IP in order to get better service (i.e., the “grease the wheels” conceptualization) has no significant association with satisfaction with the national government in Model 11.

### 3.4. Influence of IP Motivations on Life Satisfaction

We now turn to assessing the link between IP and life satisfaction. The results of ordered logit regressions on IP on the life satisfaction and the anticipated satisfaction with the future life of one's children are reported in Models 13 to 20 of Table 6. The results of these models confirm our previous findings. Overall, making IP is associated with a lower life satisfaction for respondents in Model 13. The negative effect of IP is even higher if making IP was expected or asked for (i.e., the “sand the wheels” conceptualization) in Models 16 and 20. In contrast, making IP as a customary gratitude is associated with higher life satisfaction in Models 14 and 18. In comparison, no link can be established between offering to pay IP in order to get better service (i.e., the “grease the wheels” conceptualization) in Models 15 and 19.

## 4. Discussion

Addressing the original question about the association between IP and user outcomes provides us with a novel insight. The currently popular view in the literature is that making IP has a negative effect on users' well-being [3, 9]. Most papers correlate making IP with healthcare satisfaction and have found a negative influence of IP on healthcare satisfaction [12, 54]. Our results however beg for a much more nuanced approach. As our findings suggest, only “sand the wheels” payments, when IP is asked for or felt to be required, are associated with lower satisfaction with healthcare. In sharp contrast, paying IP as a customary gratitude is associated with higher satisfaction with healthcare. In comparison, paying “grease the wheels” IP to get better services is not associated with higher satisfaction with healthcare. These findings are robust for all other measures of satisfaction that we used in this study. Thus, paying to express gratitude is linked with higher satisfaction with local and national government and higher satisfaction with life and the future life of one's children. In contrast, making IP because it was asked for or felt to be required is linked with reduced satisfaction for all the above-described measures of satisfaction. Finally, paying to get better services because one felt that IP was required is not associated with all the above-described measures of satisfaction. We can conclude therefore that the direction of association between IP and satisfaction is not universal and depends on the specific motivation for having made IP.

From a research standpoint, our findings suggest that researchers need to look beyond informal payments in general and into the specific categories that reflect the motivations for making them. Focusing on informal payments in general, rather than explicitly examining specific motivations, obscures the true outcomes of making IP. As we have demonstrated, although IP may seem to be related to lower satisfaction, our findings suggest that this is true only if respondents were asked for IP or they felt it was expected. In all other cases, making IP is associated neither with satisfaction nor with a higher level of satisfaction.

From a policy making standpoint, variation in the links between different motivations for making IP and measures of satisfaction suggests that decision-makers should put their primary focus on situations where IP are explicitly asked for or are implied by the situation and that they should differentiate this from cases of gratitude payments. If such measures are not implemented, then policy makers may unintentionally ban the behaviour that is linked with increased satisfaction with healthcare, government, and life (i.e., paying gratitude). However, differentiating between different types of IP payments may present a genuine dilemma for agencies and decision-makers who are engaged in anticorruption practice and healthcare reform.

In terms of conceptualizing IP as a cultural phenomenon which leads to positive user's outcomes, our results are in line with previous findings [12, 33, 34]. The authors of these studies suggest that giving cash to gifts to healthcare personnel is considered by users as consistent with beliefs about norms of giving and reciprocity. Our findings about the positive influence of IP as a cultural phenomenon are also in line with previous literatures which suggest that even though large-scale corruption schemes are commonly criticized, IP given to healthcare personnel are not necessarily conceptualized by users as illegal corruption and do not have negative undertone [40–43].

On the other hand, in terms of conceptualizing IP as a “grease the wheels” phenomenon, we cannot confirm the results of previous studies which suggest that such IP can improve their satisfaction [2, 45–47]. Association between “grease the wheels” payments and user's outcomes in our estimations is not positive but not statistically significant. There are three main reasons why our study cannot establish significant association between “grease the wheels” IP and users' outcomes. First, users may experience lower satisfaction even if they received better and faster services due to “grease the wheels” payments because they paid for services which they expected to be delivered for free. In other words, they may feel dissatisfaction that they have to make IP to receive higher quality and faster services since they believe that such quality and speed should be available without additional “grease the wheels” IP. Second, users could make “grease the wheels” IP to get better and faster services, but after receiving services, they may be unsatisfied with the quality and speed of services which they received [5]. Hence, they may question whether such quality and speed justify making “grease the wheels” payments.

Yet, on the other hand, in terms of conceptualizing IP as a “sand the wheels” that led to negative outcomes, our study concurs with findings of previous studies that reports that such payments are often catastrophic expenditures, especially for the poor [24]. The linkage between IP as a “sand the wheels” and negative user's outcome that we found is also in accord with other previous findings that such payments serve as the major barrier to utilization of healthcare when it is needed [8, 25, 54]. Our finding on the negative association between making IP and satisfaction with healthcare is also congruent with previous findings. Thus, Habibov [10] found that making IP in postcommunist countries is associated with a negative effect on satisfaction with public healthcare by a factor of -1.26.

In addition, the results of our study concur with the results of the recent, 2021, study by Habibov et al. [62]. The authors studied association between “grease-the-wheel,” “sand-the-wheel,” and “cultural norm” motivations for making informal payments with satisfaction in public primary, secondary, and vocational education in postcommunist countries using the same survey instrument, namely, LITS survey. Although field of research of that study was not public health, but public education, and their theoretical framework was based on a different set of assumptions than those used in our study, it is still instructive to compare their results with our results. Thus, similar to our findings, the authors reported that the association between IP and satisfaction with public education depends in a great part on the specific motivations for making IP. In line with our findings, the authors found that making IP because users were asked to by educational personnel and because such payments were expected was associated with weakened satisfaction with public education. In contradistinction, customary gratitude in form of IP was associated with increased levels of satisfaction with public education. Making IP in order to get better services was significantly associated with satisfaction. It can be concluded that difference in “grease-the-wheel,” “sand-the-wheel,” and “cultural norm” motivations for IP and satisfaction with public services exists not only in public health but also in public education. Therefore, our findings along with findings by Habibov et al. [62] suggest that more research is needed to confirm the difference in effect of “grease-the-wheel,” “sand-the-wheel,” and “cultural norm” motivations for making IP on satisfaction with public services, life satisfaction, and other well-being indicators.

At the same time, we found that the negative effect of making IP is almost equal for local and national governments. This finding suggests that turning a blind eye to “sand the wheels” payments is hardly an option since it reduces satisfaction with local and national governments. On the one hand, this finding contradicts those of Habibov et al. [64], who reported that individuals tend to blame local rather than national governments for corruption. The authors explained that healthcare is mostly managed at the local level, which helps national governments escape the blame for healthcare corruption. On the other hand, our findings that both levels of government have been blamed for corruption equally is consistent with the notion that although healthcare is managed at the local level, the major parameters and regulations of health policy and administration are established and monitored at the national level.

Another interesting finding is that the influence of making IP extends beyond proximal outcomes, such as satisfaction with healthcare, and into distal outcomes, such as life satisfaction. This finding is in line with findings of Sulemana et al. [65], which demonstrated that higher levels of informal payments have a negative effect on life satisfaction in Africa. This finding is also in line with those of Rodríguez-Pose and Maslauskaite [66] who established that happiness, in Central and Eastern European countries, is highly influenced by corruption and that the effect of corruption on happiness increased over time.

## 5. Limitations

We will be remiss without highlighting limitations of this study. First, since our data is cross-sectional, the results reflect correlation rather than causation. Second, small country samples preclude us from conducting a country-by-country analysis. Using a relatively small sample can also prevent us from accurately capturing incidents of relatively rare diseases and interventions which are frequently associated with higher propensity to make IP. Third, the LITS provides no information about the amount of IP paid and frequency of making IP, while all questions about reporting IP and getting responses as a result of reporting IP are related to the most recent incident of IP only. Finally, insofar as the LITS was not specially designed to analyse IP, the questionnaire does not allow us to differentiate between the types of health conditions (e.g., broken arm vs. cancer), healthcare facilities (e.g., primary vs. specialized), and personnel (e.g., nurses vs. technicians) who are likely to receive IP. Future research should address these specific limitations.

## 6. Conclusion

This study has revealed that it is important to distinguish between three different motivations for informal payment, namely, cultural norms, “grease the wheels,” and “sand the wheels” since they have varying associations with user outcomes. Payments that are the result of cultural norms are associated with better outcomes, while “sand the wheel” payments are associated with worsening outcomes. We found no association between making “grease the wheels” payments and outcomes. In addition, we found that these three motivations are associated with different socioeconomic correlates. Consequently, focusing on informal payments in general, rather than explicitly examining specific motivations, obscures the true outcomes of making IP.

## Figures and Tables

**Figure 1:** Flow chart of questions in LITS about making IP in public healthcare.

**Table 1:** Current health expenditure by different schemes as percentage of total health expenditures.

	Government schemes and compulsory contributory health care financing schemes	Voluntary health care payment schemes	Household out-of-pocket payment
Albania	58	0	42
Armenia	18	1	81
Azerbaijan	29	0	71
Belarus	71	2	27
Bosnia and Herzegovina	71	0	29
Bulgaria	55	1	43
Croatia	83	7	11
Czech Republic	82	3	15
Estonia	76	2	23
Georgia	37	8	56
Hungary	68	4	28
Kazakhstan	60	5	36
Kyrgyzstan	42	0	57
Latvia	56	1	43
Lithuania	67	1	32
Mongolia	64	3	32
Poland	69	8	23
Romania	78	1	21
Russia	57	3	40
Serbia	58	2	40
Slovakia	81	1	18
Slovenia	73	15	12
Tajikistan	32	2	66
Ukraine	48	3	48
Uzbekistan	45	1	55

Data is from the WHO's Global Health Expenditure database by WHO at https://apps.who.int/nha/database/Select/Indicators/en. Household out-of-pocket expenditures encompass informal payments (IP) and various legitimate fees, as detailed in Introduction.

**Table 2:** Sociodemographic and economic description of the analytical sample.

Variables	Description	Mean	Standard Deviation	Min	Max
Made informal payments in general	Made an unofficial payment or gift when using healthcare over the past 12 months: 1 = yes; 0 = no	0.18	0.38	0	1
A customary gratitude	Respondent made IP to express gratitude to healthcare personnel: 1 = yes; 0 = no	0.33	0.47	0	1
Informal payments to get better service (“grease the wheels”)	Respondent offered to pay to get better services: 1 = yes; 0 = no	0.20	0.40	0	1
Informal payment because he/she was asked to pay or felt that it was expected (“sand the wheels”)	Respondent was asked to pay by healthcare personnel or felt that IP was expected: 1 = yes; 0 = no	0.28	0.45	0	1
Satisfaction with healthcare	How satisfied with the public health service? 1 = very dissatisfied; 2 = dissatisfied; 3 = neither; 4 = satisfied; 5 = very satisfied	3.51	1.00	1	5
Satisfaction with local government	Respondent rated performance of local government: 1 = very bad; 2 = bad; 3 = neither; 4 = good; 5 = very good	3.16	0.93	1	5
Satisfaction with national government	Respondent rated performance of national government: 1 = very bad; 2 = bad; 3 = neither; 4 = good; 5 = very good	2.88	0.96	1	5
Life satisfaction	Satisfied with my life now: 1 = strongly disagree; 2 = disagree; 3 = neither disagree nor agree; 4 = agree; 5 = strongly agree	3.24	1.12	1	5
Satisfaction with children's life in future	Children will have a better life than my generation: 1 = strongly disagree; 2 = disagree; 3 = neither disagree nor agree; 4 = agree; 5 = strongly agree	3.22	1.18	1	5
*Covariates*					
Women	1 = woman; otherwise = 0	0.57	0.49	0	1
University	1 if the respondents have a Bachelor's degree or higher; otherwise = 0	0.14	0.35	0	1
Age	Age in years	48.76	17.45	18	95
Married	Married = 1 if the respondents are married; otherwise = 0	0.58	0.49	0	1
Lower level of health	1 if respondent assessed own health as bad or very bad; otherwise = 0	0.14	0.35	0	1
Number of younger children	Number of children in a household whose age is greater than 0 and less than or equal to 7	0.29	0.64	0	5
Number of older children	Number of children in a household whose age is greater than 7 and less than 17	0.35	0.71	0	7
Rural	Rural = 1 if the respondent resides in rural area; otherwise = 0	0.44	0.50	0	1
Wealth	Quintiles of family total expenditures adjusted for number of family members where 1 = to the poorest 20%of population in each country and 5 = to the wealthiest 20%of population in each country	3.00	1.42	1	5

**Table 3:** Informal payments by countries in percentage.

Country	Making informal payments	Percentage
*Eastern European countries*		
Czech Rep.	89	9.80
Estonia	67	5.36
Hungary	239	25.18
Latvia	142	11.52
Lithuania	303	24.44
Poland	69	6.59
Slovak Rep.	135	12.88
Slovenia	24	2.09
*South European countries*		
Albania	242	30.79
Bosnia and Hercegovina	158	19.39
Bulgaria	134	15.95
Croatia	72	9.07
FYR Macedonia	71	10.35
Romania	209	29.73
Serbia	98	13.26
*Countries of the former Soviet Union and Mongolia*		
Armenia	170	19.08
Azerbaijan	131	34.38
Belarus	160	17.86
Georgia	21	3.11
Kazakhstan	133	18.63
Kyrgyz Rep.	177	24.72
Moldova	238	41.75
Mongolia	96	16.52
Russia	195	21.76
Tajikistan	260	45.69
Ukraine	251	33.92
Uzbekistan	132	15.96

**Table 4:** Satisfaction with healthcare.

	Model 1	Model 2	Model 3	Model 4
Made IP in general	0.392^∗∗∗^ (0.014)			
Customary gratitude		3.455^∗∗∗^ (0.245)		
Offered to pay to get better service (“grease the wheels”)			0.911 (0.068)	
Asked to pay or felt that IP was expected (“sand the wheels”)				0.379^∗∗∗^ (0.024)
Women	1.110^∗∗∗^ (0.029)	1.144^∗^ (0.071)	1.150^∗^ (0.071)	1.186^∗∗^ (0.074)
Age	1.007^∗∗∗^ (0.001)	1.004 (0.002)	1.005^∗^ (0.002)	1.005^∗^ (0.002)
Married	0.968 (0.027)	1.059 (0.071)	1.006 (0.067)	1.027 (0.068)
University	1.060 (0.041)	1.014 (0.092)	1.064 (0.096)	1.031 (0.093)
Number of older children	0.992 (0.020)	0.980 (0.043)	0.987 (0.043)	0.970 (0.042)
Number of younger children	1.028 (0.023)	1.063 (0.054)	1.089 (0.055)	1.087 (0.055)
Wealth	0.979^∗^ (0.010)	0.969 (0.023)	0.977 (0.023)	0.963 (0.022)
Rural	1.137^∗∗∗^ (0.032)	1.156^∗^ (0.078)	1.164^∗^ (0.078)	1.186^∗^ (0.079)
Lower level of health	0.639^∗∗∗^ (0.024)	0.652^∗∗∗^ (0.056)	0.632^∗∗∗^ (0.053)	0.645^∗∗∗^ (0.055)
Country dummies included	YES	YES	YES	YES
*N*	22,529	3807	3807	3807
Log likelihood	-27653.14	-5117.49	-5276.90	-5159.74
McKelvey & Zavoina *R*^2^	0.122	0.146	0.067	0.125
LR chi^2^	2675.78^∗∗∗^	569.01^∗∗∗^	250.22^∗∗∗^	484.50^∗∗∗^

Standard errors in parentheses: ^∗^*p* < 0.05, ^∗∗^*p* < 0.01, and ^∗∗∗^*p* < 0.001.

**Table 5:** Satisfaction with local and national governments.

	Local government				National government			
	Model 5	Model 6	Model 7	Model 8	Model 9	Model 10	Model 11	Model 12
Made IP in general	0.665^∗∗∗^ (0.024)				0.675^∗∗∗^ (0.025)			
Customary gratitude		1.643^∗∗∗^ (0.116)				1.704^∗∗∗^ (0.128)		
Offered to pay to get better service (“grease the wheels”)			0.889 (0.070)				0.893 (0.073)	
Asked to pay or felt that IP was expected (“sand the wheels”)				0.708^∗∗∗^ (0.046)				0.685^∗∗∗^ (0.048)
Socioeconomic covariates included^1^	Yes	Yes	Yes	Yes	Yes	Yes	Yes	Yes
Country dummies included	Yes	Yes	Yes	Yes	Yes	Yes	Yes	Yes
*N*	21,028	3,599	3,599	3599	19,715	3,313	3,313	3,313
Log likelihood	-25,889.09	-4,609.35	-4,633.12	-4,620.22	-23,869	-3,966.83	-3,991.32	-3,977.41
McKelvey & Zavoina *R*^2^	0.130	0.166	0.153	0.160	0.233	0.276	0.276	0.284
LR chi^2^	2,739.98^∗∗∗^	602.42^∗∗∗^	554.88^∗∗∗^	580.68^∗∗∗^	4,767.30^∗∗∗^	1,015.55^∗∗∗^	966.57^∗∗∗^	994.38^∗∗∗^

Standard errors in parentheses: ^∗^*p* < 0.05, ^∗∗^*p* < 0.01, and ^∗∗∗^*p* < 0.001. ^1^The same socioeconomic covariates as in Table 2.

**Table 6:** Life satisfaction.

	Satisfaction with life now				Children will be happier than my generation			
	Model 13	Model 14	Model 15	Model 16	Model 17	Model 18	Model 19	Model 20
Made IP in general	0.895^∗∗^ (0.030)				0.987 (0.035)			
Customary gratitude		1.356^∗∗∗^ (0.093)				1.640^∗∗∗^ (0.117)		
Offered to pay to get better service (“grease the wheels”)			1.063 (0.081)				0.872 (0.069)	
Asked to pay or felt that IP was expected (“sand the wheels”)				0.738^∗∗∗^ (0.047)				(0.047)
Socioeconomic covariates included^1^	Yes	Yes	Yes	Yes	Yes	Yes	Yes	Yes
Country dummies included	Yes	Yes	Yes	Yes	Yes	Yes	Yes	Yes
*N*	22,392	3,778	3,778	3,778	20,667	3,498	3,498	3,498
Log likelihood	-29,538.17	-5,122.78	-5,132.42	-5,121.16	-28,502.26	-4,814.12	-4,836.84	-4,825.84
McKelvey & Zavoina *R*^2^	0.189	0.186	0.182	0.187	0.176	0.174	0.162	0.167
LR chi^2^	4,445.19^∗∗∗^	749.1^∗∗∗^	729.81^∗∗∗^	752.34^∗∗∗^	3909.16^∗∗∗^	626.15^∗∗∗^	580.73^∗∗∗^	602.73^∗∗∗^

Standard errors in parentheses: ^∗^*p* < 0.05, ^∗∗^*p* < 0.01, and ^∗∗∗^*p* < 0.001. ^1^The same socioeconomic covariates as in Table 2.

## Data Availability

Data is available at http://www.ebrd.com.

## Abbreviations

IP: Informal payments
LITS: Life in Transition Survey
EBRD: European Bank for Reconstruction and Development.
